The article "Research on Effects of Oropharyngeal Aspiration on Incidence of Ventilator-Associated Pneumonia in Patients with Cerebral Hemorrhage in ICU" was retracted in 2023. Reason: compromised peer review.

# Research on Effects of Oropharyngeal Aspiration on Incidence of Ventilator-Associated Pneumonia in Patients with Cerebral Hemorrhage in ICU

**DOI:** 10.1155/2022/6433666

**Published:** 2022-01-18

**Authors:** Linli Qi, Xiaoxia Guo, Chunyan Nie, Xin Lv, Miao Zhang

**Affiliations:** ^1^The 2nd Ward of Microinvasive Neurosurgery, The Fourth Affiliated Hospital of Harbin Medical University, Harbin 150000, China; ^2^Department of Competent Nursing, The Fourth Affiliated Hospital of Harbin Medical University, Harbin 150000, China; ^3^Department of Elderly Ward, The Fourth Affiliated Hospital of Harbin Medical University, Harbin 150000, China

## Abstract

Cerebral hemorrhage is a kind of intracranial hemorrhage caused by nontraumatic vascular rupture of the cerebral parenchyma, which is a common cerebrovascular disease with a high disability rate and mortality. This study aimed to explore the effects of oropharyngeal aspiration in reducing ventilator-associated pneumonia in patients with cerebral hemorrhage in ICU. In this study, 96 patients with cerebral hemorrhage were selected as the subjects. They received surgical treatment, and then they were transferred into ICU of Fourth Affiliated Hospital of Harbin Medical University from December 2019 to March 2020. The patients were randomly divided into intervention group and control group, with 48 in each group. The intervention group received periodic oropharyngeal aspiration, while the control group received routine nursing measures. After the intervention, the incidence of ventilator-associated pneumonia and the positive rate of amylase *α*-trachea cannula specimens were recorded and compared between the two groups. After the intervention, the incidence of ventilator-associated pneumonia was 14.89% in the intervention group and 39.58% in the control group, with a statistically significant difference. And, the *α*-amylase positive rate, mechanical ventilation time, and ICU care duration of endotrachea cannula specimens in the intervention group were significantly lower than those in the control group. In conclusion, oropharyngeal aspiration can effectively reduce the incidence of ventilator-associated pneumonia after cerebral hemorrhage and shorten mechanical ventilation and ICU care duration. It promotes the rehabilitation of patients.

## 1. Introduction

Cerebral hemorrhage is a kind of intracranial hemorrhage caused by nontraumatic vascular rupture of cerebral parenchyma, which is a common cerebrovascular disease with high disability rate and mortality [1, 2]. Currently, minimally invasive removal of intracranial hematoma is a common method for treating patients with cerebral hemorrhage, which can effectively alleviate clinical symptoms [3]. However, patients are usually in coma early after operation without autonomous respiration, so they need a ventilator assisting ventilation [4]. Mechanical ventilation will cause many complications, the most serious of which is ventilator-associated pneumonia. According to previous studies, 30% to 65% of patients with cerebral hemorrhage in ICU have ventilator-associated pneumonia, which is one of the main causes of death in the first month after surgery for cerebral hemorrhage. It accounts for about 30% of mortality 30 days after surgery [5]. Furthermore, ventilator-associated pneumonia can result in prolonged mechanical ventilation and hospital stay in patients in ICU. Intervention of standardized postoperative nursing measures reduced the incidence of ventilator-associated pneumonia, but did not completely address risk factors.

The article "Research on Effects of Oropharyngeal Aspiration on Incidence of Ventilator-Associated Pneumonia in Patients with Cerebral Hemorrhage in ICU" was retracted in 2023. Reason: compromised peer review.

Microaspiration of secretions is a common cause of ventilator-associated pneumonia in patients in ICU. It is defined as that the patient involuntarily inhales the oropharyngeal secretions around the trachea cannula into the tracheal intubation [6, 7]. A number of studies have detected *α*-amylase in trachea cannula in patients with ventilator-associated pneumonia, indicating that the patients had microaspiration of secretions [8–10]. The results of the study by Weiss et al. showed that *α*-amylase level was increased in the microaspiration of secretions obtained by bronchoalveolar lavage within 72 h after trachea cannula. This increase was related to trachea cannula microaspiration of secretions, which could be used to predict ventilator-associated pneumonia. *α*-Amylase is a biomarker of human oropharyngeal microaspiration of secretions, which does not exist in the lungs. Evidence-based data shows that *α*-amylase is a predictor of trachea cannula microaspiration of secretions leakage and ventilator-associated pneumonia in mechanically ventilated populations [11]. Moreover, studies have reported that *α*-amylase levels in the lungs of patients with ventilator-associated pneumonia are also significantly higher than those in patients without ventilator-associated pneumonia [12]. Nasal and oral cavity secretions accumulate above the cuff of tracheal catheter and below the glottis in patients with cerebral hemorrhage in ICU receiving mechanical ventilation. And, the *α*-amylase positive rate, mechanical ventilation time, and ICU care duration of endotrachea cannula specimens in the intervention group were significantly lower than those in the control group. Therefore, *α*-amylase was used as a biomarker to explore the effect of targeted intervention to reduce trachea cannula microaspiration of secretions by oropharyngeal aspiration on ventilator-associated pneumonia in patients with cerebral hemorrhage in ICU.

The article "Research on Effects of Oropharyngeal Aspiration on Incidence of Ventilator-Associated Pneumonia in Patients with Cerebral Hemorrhage in ICU" was retracted in 2023. Reason: compromised peer review.

## 2. Research Subjects and Methods

### 2.1. Participants and Recruitment Process

From December 1, 2019, to March 31, 2020, patients with cerebral hemorrhage were selected as the subjects. They received minimally invasive removal of intracranial hematoma and were transferred into ICU of Fourth Affiliated Hospital of Harbin Medical University. Inclusion criteria: (1) patients who were diagnosed with cerebral hemorrhage by cranial CT or MRI and clinical evaluation, with the amount of bleeding ranging 15 to 160 ml; (2) patients who were in accordance with the surgical indications for cerebral hemorrhage; (3) patients transferred to ICU after surgical treatment; (4) patients whose trachea cannula was expected to continue for more than 36 hours. Exclusion criteria: (1) patients with pontine hemorrhage; (2) patients under rescue mechanical ventilation therapy (high-frequency oscillator ventilation or in vitro membrane oxygenation); (3) patients with pupil dilation; (4) patients with organ failure or organ dysfunction; (5) patients with contraindications to intervention (e.g., oropharyngeal injury). With the approval of the ethics review committee, researchers screened 107 eligible patients based on inclusion criteria. Because patients in ICU cannot sign their own informed consent, researchers explained this study and its potential risk benefits to the patients' families. After ensuring that the family understood the contents of informed consent, all the family members of patients who volunteered to join the study signed the informed consent. In this study, 96 patients' families signed the informed consent.

### 2.2. Random Grouping

The researchers input subjects' names into Excel documents by computer and used the random number function to generate random numbers following each patient's name. According to the numbers, the first 50% of the patients were included in the intervention group, and the last 50% of the patients were included in the control group, with 48 patients in each group.

### 2.3. Intervention Group

#### 2.3.1. Intervention Programming

According to the results of the literature review, the intervention plan was decided. A 21 cm oropharyngeal aspiration catheter was used to aspirate the oropharynx around trachea cannula every 4 h in the intervention group. During aspiration, the oropharyngeal aspiration catheter was positioned to reach both sides of the oral cavity and oropharynx. The nurse uses standard aspiration negative pressure to perform aspiration in real-time. The aspiration stops when no secretions can be heard or seen. Intervention will be stopped when the patient has the following conditions: (1) tracheal intubation was removed according to doctor's advice; (2) transferred out of ICU according to doctor's advice; (3) treat with tracheotomy; (4) included into the study for 15 days. Intervention was set to last for 15 days because patients in this study were transferred out of ICU 15 days after being included.

The article "Research on Effects of Oropharyngeal Aspiration on Incidence of Ventilator-Associated Pneumonia in Patients with Cerebral Hemorrhage in ICU" was retracted in 2023. Reason: compromised peer review.

#### 2.3.2. Intervention Implementing

The research group consisted of researchers and 4 ICU nurses. Researchers trained 4 ICU nurses for 3 hours to ensure uniformity of intervention before the study started, including aspiration duration, depth, frequency, cycle, and stop aspiration standard, with methods of viewing a video, explaining on PPT, and simulation operation. After training, researchers issued intervention manuals and intervention records containing the training content for the intervention implementers to use. During the intervention, 4 nurses were assigned to different duty periods. During their duty, nurses recorded the time and frequency of aspiration in patients on the intervention record book and handed over to the subsequent nurses according to the average duration of 45.2 ± 3.7 s in this study.

### 2.4. Control Group

Nurses cleaned the patient's oropharyngeal microaspiration of secretions with saline cotton balls every 4 h and cleaned the patient's oropharynx with oral antimicrobial agents and toothbrushes every 12 h.

### 2.5. Data Collection

General demographic data and disease-related information were collected at the patients' admittance, including age and sex in general demographic data, history of chronic obstructive pneumonia, history of chronic heart disease, location of cerebral hemorrhage, and amount of cerebral hemorrhage in disease-related information.

Outcome indexes for this study included the number of cases of ventilator-associated pneumonia, the percentage of *α*-amylase positive in trachea cannula specimens, the mean value of *α*-amylase, IL-6, IL-8, PSP, NE, su-PAR, IL-35, soluble triggering receptor expressed on myeloid cell-1 (sTREM-1), penetrant-3 (PTX-3), procalcitonin (PCT), ICU care duration, and mechanical ventilation time in trachea cannula specimens. The number of cases of ventilator-associated pneumonia was collected immediately after intervention. Ventilator-associated pneumonia was diagnosed by doctors according to the diagnostic criteria as follows: clinical indexes: (1) paroxysm after 48 h of ventilation; (2) intrapulmonary infiltration shadows or new inflammatory lesions compared with the chest radiographs before mechanical ventilation; (3) signs of pulmonary consolidation; (4) body temperature above 38.8°C without other known causes; (5) purulent sputum new or sputum characteristics change and increased respiratory secretions; (6) new or deteriorating cough or dyspnea or shortness of breath; etiological indexes: (1) aleucocytosis (<4000 WBC/mm^3^) or leucocytosis (12,000 WBC/mm^3^); (2) bacterial culture of endotracheal aspirate or bronchoalveolar lavage fluid was positive [13]. The researchers immediately sucked the secretions through the endotracheal tube with a disinfectant pipette to obtain the endotracheal intubation specimen. The content of *α*-amylase was measured as an important biological index to evaluate the microaspiration of secretions. Trachea cannula specimens were stored in a −20°C container until determination was performed by inspection personnel. The *α*-amylase values of each trachea specimen were recorded as U/L, 392 U/L was regarded as the standard of microabsorption of microaspiration of secretions [14]. As indexes of mediating and activating individual immune and inflammatory responses, IL-6 and other cytokines increased in the presence of individual infection. After intervention, researchers extracted the blood of patients to detect the level of serum inflammatory response factors. In addition, patients' ICU care duration and mechanical ventilation time were recorded with an electronic medical record system.

The article "Research on Effects of Oropharyngeal Aspiration on Incidence of Ventilator-Associated Pneumonia in Patients with Cerebral Hemorrhage in ICU" was retracted in 2023. Reason: compromised peer review.

### 2.6. Data Analysis

SPSS 24.0 was used for statistical data description and analysis. The measurement data were expressed by mean and standard deviation, and the counting data were expressed by frequency and percentage. The comparability of demographic and disease-related baseline data between two groups was compared with chi-square test or independent sample *t*-test. Chi-square test was used to evaluate the incidence of ventilator-associated pneumonia in both groups. And, the independent sample *t*-test and chi-square test were also used to calculate the percentage of secretory microabsorbent positive samples between two groups and the difference of *α*-amylase average over time. The difference ICU care duration, mechanical ventilation time, and inflammatory response index between two groups were evaluated with the independent sample *t*-test. All data analysis results were statistically significant in bilateral *P* < 0.05.

## 3. Results

### 3.1. Comparison of Baseline Data Scores between Two Groups

96 patients were included in the intervention. There were 48 patients in the control group, with 26 males and 22 females, aged 49∼76 years old, with the average age of (65.72 ± 3.95) years old. Of which, there were 21 cases of brain lobe hemorrhage, 18 cases of putamen hemorrhage, 9 cases of thalamus hemorrhage, 1 case of chronic heart disease, and 2 cases of chronic obstructive pulmonary disease. 48 patients were included in the intervention group, with 25 males and 23 females, aged 55∼79 years old, with the average age of 66.16 ± 4.38 years old. Of which, there were 20 cases of brain lobe hemorrhage, 22 cases of putamen hemorrhage, 6 cases of thalamus hemorrhage, 1 case of chronic obstructive pulmonary disease, and 3 cases of chronic heart disease. There was no significant difference in age, sex ratio, and location between two groups. Chronic obstructive pulmonary disease and chronic cardiac disease are risk factors that increase the risk of ventilator-associated pneumonia, with no significant difference in the prevalence of chronic obstructive pulmonary disease and chronic heart disease between two groups. The above results showed that the baseline data of the two groups are consistent, with comparability.

The article "Research on Effects of Oropharyngeal Aspiration on Incidence of Ventilator-Associated Pneumonia in Patients with Cerebral Hemorrhage in ICU" was retracted in 2023. Reason: compromised peer review.

### 3.2. Comparison of Incidence of Ventilator-Associated Pneumonia and Changes with Time after Intervention between Two Groups

According to chi-square test, the incidence of ventilator-associated pneumonia was significantly different between two groups after intervention, and the incidence of patients in the intervention group was significantly lower than that in the control group (Table 1).

### 3.3. Comparison of Percentage of *α*-Amylase Positive Specimens and Average Content of *α*-Amylase after Intervention between Two Groups

The results of chi-square test showed that the percentage of positive specimens in patients of the control group was significantly higher than that in the intervention group (Table 2). The results *t* independent samples indicated that *α*-amylase in the control group was significantly higher than that in the intervention group (Table 3).

### 3.4. Comparison of Difference of Inflammatory Response Indexes after Intervention between Two Groups

The results of independent sample *t* test showed that IL-6, IL-8, PSP, NE, su-PAR, IL-35, sTREM-1, PTX-3, and PCT levels of patients in the control group was higher than that in the intervention group (*P* < 0.05), as shown in Table 4.

### 3.5. Comparison of the Mean Mechanical Ventilation Time and ICU Care Duration after Intervention between Two Groups

Both mechanical ventilation time and ICU care duration in the intervention group were significantly lower than those in the control group, as shown in Table 5.

## 4. Discussion

Nasal and oral cavity secretions accumulate above the cuff of the tracheal catheter and below the glottis in patients with cerebral hemorrhage in ICU receiving mechanical ventilation [15, 16]. In patients with endotracheal intubation, opening oral cavity, and airway easily can cause pathogenic bacteria colonizing secretions that collect in the oropharynx. If leakage occurs around the cuff of trachea catheter, the microaspiration of secretions containing pathogenic bacteria around the oropharynx will spread along trachea cannula to the lower respiratory tract of patients, resulting in ventilator-associated pneumonia [17]. Moreover, studies have reported that *α*-amylase levels in the lungs of patients with ventilator-associated pneumonia are also significantly higher than those in patients without ventilator-associated pneumonia [12]. Regular oropharyngeal aspiration can remove some microaspiration of secretions of oropharynx in time, prevent bacterial colonization of oropharynx, and reduce the risk of ventilator-associated pneumonia caused by microaspiration of oropharynx microaspiration of secretions [18–20]. Although oropharyngeal aspiration may have clinical benefits for patients in need of mechanical ventilation, there is no nursing management standard ICU ventilator-associated pneumonia in patients with trachea cannula. At the same time, there are great differences in oropharyngeal aspiration tools, frequency, and location in reducing ventilator-associated pneumonia [21–23]. On the basis of synthesizing and analyzing the existing intervention research evidence, this study used a 21 cm oropharyngeal aspiration catheter to carry out periodic oropharyngeal aspiration every 4 h in order to reduce the incidence of ventilator-associated pneumonia in patients with cerebral hemorrhage in ICU [24, 25]. The results showed that the incidence of ventilator-associated pneumonia in patients receiving regular oropharyngeal aspiration was significantly lower than that in patients without intervention, and the risk of ventilator-associated pneumonia in the control group was significantly higher than that in the intervention group, revealing that oral aspiration could significantly reduce the incidence and risk of ventilator-associated pneumonia.

The article "Research on Effects of Oropharyngeal Aspiration on Incidence of Ventilator-Associated Pneumonia in Patients with Cerebral Hemorrhage in ICU" was retracted in 2023. Reason: compromised peer review.

Meanwhile, in this study, *α*-amylase sample of ventilation duct was positive, which has been confirmed as another significant risk factor for ventilator-associated pneumonia. Compared with patients in the control group, *α*-amylase content and positive rate of patients in the intervention group were significantly lower than those in the control group. Through the analysis of serum inflammatory factors, the level of serum inflammatory factor was significantly lower than that of the control group. The results supported the hypothesis of this study, namely, regular oropharyngeal aspiration can remove the accumulated oropharyngeal secretions in a timely manner and reduce microaspiration of secretions, thus reducing the possibility of oropharyngeal pathogens entering the trachea through catheterization and causing ventilator-associated pneumonia. Previous retrospective studies showed that, without intervention, *α*-amylase positive rates in endotracheal intubation samples of patients with mechanical ventilation ranged from 68.6% to 77.4% [26]. The positive rate was similar to that of *α*-amylase in trachea cannula samples in the control group, but significantly higher than that in the intervention group, showing that oropharyngeal aspiration can effectively reduce microaspiration of secretions microaspiration by regularly removing oropharynx accumulated microaspiration of secretions. The decrease of microaspiration of secretions aspiration may reduce the probability that oropharyngeal pathogens enter patient's lungs through tracheal catheter, leading to pulmonary inflammation. When the individual is infected by bacterial invasion, the inflammatory factor is activated and its expression will be significantly increased and released into the blood, leading immune cells to identify and eliminate pathogens. The results of previous studies showed that, after ventilator-associated pneumonia, the systemic and local inflammatory responses were aggravated, and the levels of inflammatory factors, such as IL-6, IL-8, sTREM-1, PTX-3, and PCT, in serum increased significantly [27]. The serum immune factor level in the intervention group was lower than that, in the control group, which cannot confirm the causal relationship between the difference of inflammatory factors between two groups and the decrease of oropharyngeal pathogens entering the lower respiratory tract caused by oropharyngeal aspiration. However, it shows that oropharyngeal aspiration can reduce the possibility of infection caused by oropharyngeal pathogens entering the lower respiratory tract through the trachea. The hypothesis of this study can be further confirmed by comparing oropharyngeal pathogens with pulmonary pathogens through bacterial etiological analysis.

## 5. Conclusion

Furthermore, compared with the control group, the mechanical ventilation time and ICU care duration in the intervention group were significantly lower than those in the control group, suggesting that the effective management of ventilator-associated pneumonia can promote the rehabilitation of lung function and physical function, shorten the mechanical ventilation time and ICU care duration, and reduce the cost of treatment.

Based on the literature review of the intervention time, intervention frequency, and intervention tool selection of oropharyngeal aspiration in patients transferred to ICU after cerebral hemorrhage, the intervention program was established to test the intervention effect, which provided a reference for nursing staff to prevent pulmonary infection, advance the rehabilitation of patients, and shorten the mechanical ventilation time. Pulmonary infection is a common postoperative complication, which seriously endangers the health of patients with a high cost of treatment. Therefore, the oropharyngeal aspiration proposed in this study is an easy-to-operate nursing intervention based on evidence, with certain clinical significance to improve the rehabilitation effect of patients with cerebral hemorrhage in ICU.

The article "Research on Effects of Oropharyngeal Aspiration on Incidence of Ventilator-Associated Pneumonia in Patients with Cerebral Hemorrhage in ICU" was retracted in 2023. Reason: compromised peer review.

## Figures and Tables

**Table 1:** Comparative of incidence of ventilator-associated pneumonia *n *(%).

Group	Ventilator pneumonia		*n*	Chi-square	*P*
	Yes	No			
Intervention group	7 (14.58)	41 (85.42)	48	7.596	0.006
Control group	19 (39.58)	29 (60.42)	48		

**Table 2:** Differences in positive specimen rates between two groups.

Group	Positive	Negative	*n*	Chi-square	*P*
Intervention group	22 (45.83)	26 (54.17)	48	9.895	0.002
Control group	37 (77.08)	11 (60.42)	48		

**Table 3:** Difference of *α*-amylase content in specimens between two groups ($\bar{\text{X}}$ ± SD).

	Intervention group	Control group	*t*	*P*
*α*-Amylase content (U/L)	17982 ± 16643	10569 ± 11838	2.515	0.014

**Table 4:** Differences in levels of validation response indexes after intervention between two groups ($\bar{\text{X}}$ ± SD).

Inflammatory indexes	Intervention group (*n* = 48)	Control group (*n* = 48)	*t*	*P*
IL-6 (ng/L)	247.67 ± 25.93	279.36 ± 25.48	6.039	＜0.001
IL-8 (pg/ml)	325.83 ± 32.19	350.74 ± 35.72	3.589	0.001
PSP (ng/ml)	40.90 ± 8.16	49.98 ± 9.63	4.984	＜0.001
NE (*μ*g/L)	153.77 ± 34.57	207.24 ± 38.37	7.713	＜0.001
su-PAR (ng/ml)	8.21 ± 2.15	12.06 ± 2.42	8.240	＜0.001
IL-35 (pg/ml)	30.96 ± 4.77	37.78 ± 4.85	6.946	＜0.001
sTREM-1 (pg/ml)	174.13 ± 26.32	188.53 ± 29.59	2.519	0.013
PTX-3 (ng/ml)	14.25 ± 6.42	21.39 ± 8.74	4.562	＜0.001
PCT (*μ*g/L)	0.57 ± 0.20	0.79 ± 0.26	9.833	＜0.001

**Table 5:** Comparison of mechanical ventilation time and ICU care duration after intervention between two groups ($\bar{\text{X}}$ ± SD).

Group	Number of cases (cases)	Mechanical ventilation time (Day)	ICU care duration (Day)
Intervention group	48	5.16 ± 1.69	7.20 ± 2.65
Control group	48	9.80 ± 1.20	10.68 ± 2.92
*t*		15.509	6.114
*P*		0.000	0.000

## Data Availability

The datasets used and/or analyzed during the present study are available from the corresponding author on reasonable request.
